RETRACTED

# Optimization of Choreography Teaching with Deep Learning and Neural Networks

**DOI:** 10.1155/2022/7242637

**Published:** 2022-07-31

**Authors:** Qianling Zhou, Yan Tong, Hongwei Si, Kai Zhou

**Affiliations:** ^1^School of Music and Dance, Hunan Women's University, Changsha 410004, Hunan, China; ^2^School of Music, South China Normal University, Guangzhou 510631, Guangdong, China; ^3^Department of the History of Science, Tsinghua University, Beijing, China; ^4^School of Social Development and Management, Hunan Women's University, Changsha 410004, Hunan, China

## Abstract

To improve the development level of intelligent dance education and choreography network technology, the research mainly focuses on the automatic formation system of continuous choreography by using the deep learning method. Firstly, it overcomes the technical difficulty that the dynamic segmentation and process segmentation of the automatic generation architecture in traditional choreography cannot achieve global optimization. Secondly, it is an automatic generation architecture for end-to-end continuous dance notation with access to temporal classifiers. Based on this, a dynamic time-stamping model is designed for frame clustering. Finally, it is concluded through experiments that the model successfully achieves high-performance movement time-stamping. And combined with continuous motion recognition technology, it realizes the refined production of continuous choreography with global motion recognition and then marks motion duration. This research effectively realizes the efficient and refined production of digital continuous choreography, provides advanced technical means for choreography education, and provides useful experience for school network choreography education.

## 1. Introduction

Dance is a performance art based on human activities, expressing dancers' emotions and spiritual desires through the body language. Traditional dance is related to the historical and geographical environment, human and geographical conditions, and other reasons. It represents the most urgent voice of human beings in the situation at that time, as well as the praise and pursuit of a better life. Before there was no recording equipment, the inheritance of traditional dance mostly relied on oral and personal teaching and was easily misrepresented and lost due to various external factors. After the widespread use of photography and video technology, although pictures and videos have become the main recording forms of traditional dance and body art, they still cannot overcome the practical problem of accurate preservation of traditional dance. The picture is two-dimensional (2D) information content, but the dancing dynamic is essentially the dynamic of the body in the three-dimensional (3D) space. The single picture recording will lead to the loss of depth information so that the viewer lacks the 3D spatial experience of the dancing dynamic. The shooting of high-definition photos also requires huge human and financial resources, and the work efficiency is low.

RETRACTED

Choreography has now become an important part of the art department of various colleges and the art discipline of comprehensive universities. Due to the development of computer technology, humans have invented various machine learning (ML) algorithms to generate dance movements by dynamically capturing information [1]. Hidden Markov model (HMM) is also used to generate dance movements. As early as 2005, a new model nonparameter hierarchy hidden Markov model (NPHHMM) was born, which was a hierarchical HMM with nonparametric output density [2]. This model can be applied to the manufacture of reproducible motion engines for learning and human motor abilities. Some scholars have also considered combining acoustic analysis with text [3] and proposed a scheme to obtain 3D virtual humans from sound information by using the inferred acoustic and semantic features of the human language. By studying the rhythm of acoustic information and correlating it with related lexical meanings, vivid virtual facial expressions and dynamics are formed [4], such as head movements, binocular saccades, gestures, blinks, and gazes. The researchers confirmed that their algorithm is far superior to traditional algorithms that generate virtual humans only through speech rhythm [5].

The use of computer technology to automatically generate choreography is the research of great practical significance and necessity, because the existence of motion capture technology has replaced the traditional naked-eye observation technology, providing a bridge for automatic switching between real dance and choreography records. A choreography model and a choreography teaching semi-supervised system based on neural networks (NNs) are proposed. According to the human skeleton characteristics with vectors, and on the basis of combining the position characteristics of human joints and skeleton vector characteristics, the skeleton topology is innovatively encoded by the adjacency matrix. Through the multi-NNs model, correlation modeling of spatiotemporal signals can effectively enhance the recognition accuracy of human motion in the model. It provides a theoretical basis for choreography education and improves the level of choreography education and the effectiveness of teaching work. It also provides a useful experience and reference for choreography education in school and is of great significance to the inheritance and protection of traditional dance.

RETRACTED

## 2. Methods

### 2.1. Commonly Used Dance Notation Database in Choreography Teaching and Its Structure

As a scientific and vivid human action symbol memory system, dance notation has been widely used in the global dance world, since it was first proposed, and has played a vital role in the field of dance education. A complete choreography is mainly composed of two parts: vertical staff and choreographic characters [6]. Commonly used choreography is shown in Figure 1.

In Figure 1(a), the hidden action time axis in the dance notation from the bottom to the top and action symbols are arranged from the bottom to the top according to the time sequence, so people can read the dance notation of each page from the bottom to the top.  Figure 1(b) represents the uniform walking process with the left and right legs interacting; Figure 1(c) shows two postures with different durations of the right knee movements; Figure 1(d) records the movements of the hand, the left arm, and the right hand. As for the movement of the support part of the body, it is necessary to analyze the dynamic change process of the center of gravity of the body and the limbs, which is the key point in the analysis of the body movement. The display of dance notation during posture conversion is displayed in Figure 2 [7].

Figure 2 denotes the movements of the two legs. Although the moving positions in the horizontal direction are both right, they are decomposed into different choreography symbols because of the different processes of changing the center of gravity. The analysis of static dance movements is relatively simple. Since the related technologies are relatively complete, this chapter focuses on the dynamic analysis of the support part of the lower limb movement and leg movements in the discussion of the automatic generation algorithm of choreography [8].

Motion capture technology refers to the information technology that tracks and records the movement track or posture of moving objects in the real 3D space and saves and reconstructs the recorded sports status information on computer equipment [9]. The motion capture technology in film and television products is expressed in Figure 3.

In Figure 3, this technology is widely used in animation and film and television creation, virtual reality (VR), human-computer interaction (HCI), and so on. The most common base video handler (BVH) format is used to save motion capture data. This format defines the human skeleton as a tree model composed of 18 joints. The skeletal node model of the human is demonstrated in Figure 4 [10].

RETRACTED

In Figure 4, the red dots represent the motion capture data area, starting with a keyword. First, the total number of frames of the motion capture data in this segment is written out, and marked with the keyword. Then, the basic motion data of each frame is provided according to the hierarchical order of the definition area, including the corresponding spatial displacement of the root node, which is displayed in the form of a 3D coordinate system. There is a specific continuity between element actions involved in continuous human motion, but the traditional architecture cannot take this into account, so it cannot provide the global optimal solution of the continuous action sequence [11]. The framework for automatic generation of continuous dance notation by the connectionist temporal classification (CTC) is exhibited in Figure 5.

In Figure 5, a series of choreography sessions are manually formed by CTC technology. Its main function in the manual formation architecture of continuum is the dynamic detection of each frame of the inputting continuous action in the deep neural network (DNN). The results are decoded and transcribed into the symbolic order of the best-choreographed dance notation [12].

### 2.2. Choreography Model Based on NNs

The peculiar structure of convolutional neural networks (CNN) makes it show a better performance in technologies, such as speech recognition and image processing [13]. The most commonly used 2D CNN treats small parts of the image as inputs to the lower layers of the hierarchy, and data is passed to the deeper layers in turn. This method processes information through a one-dimensional CNN, which is used to obtain more expressive high-level information from the spatial level [14]. The weights of the same convolution kernel are shared on the same channel, and different convolution kernels can extract different features. For an input vector *X* ∈ *R*^*N*×*M*^ and filter *W* ∈ *R*^*n*×*m*^, the calculation of the convolution between the two is shown in the following equation:

(1) $$\begin{array}{c} H_{ij}=\sum_{k}^{m}\sum_{l}^{n}W_{kl}\cdot X_{i-k+1,j-l+1}. \end{array}$$

In (1), *H* is the equation of the convolution calculation, *X* is the input vector, *W* is the filtered signal, *m, k, n* are the convolution kernels, and *i, j* are the numbers of the convolution kernels [15]. The algorithm diagram of CNN is expressed in Figure 6.

In Figure 6, feature extraction is mainly performed by convolutional layers in CNN. The convolutional layer contains many convolution kernels, which can be used as 2D filters, and each convolution kernel has corresponding connection weights and biases [16]. Each operation can obtain an activation value, and the weights of multiple convolution kernels are shared on a channel, so different convolution kernels can extract different features.

RETRACTED

Gated recurrent unit (GRU) is a variant of the recurrent neural network (RNN), which introduces a neural module architecture on the cornerstone of traditional network systems. It can effectively overcome the long-term memory that RNN cannot carry out, and the phenomenon of exploding gradient or gradient descent occurs in the process of back-propagation of information [17]. Compared with another RNN variant, the “gated” unit in the long short-term memory (LSTM), because there is one less gate structure inside the GRU, the parameters involved are smaller, the training time is shorter, and higher computational efficiency and superior characteristics are obtained. Therefore, building a computer network with GRU neural units to process time series data is a more efficient option. The internal structure and the pruning algorithm of GRU are shown in Figure 7.

Figure 7 denotes the gate structure of GRU. GRU combines the unit state and the hidden state in LSTM into an independent hidden state *h*, and modifies the following two gate structures: an update gate, as shown in *t*. Its function is similar to the input gate and the forget gate in LSTM, which can be used to restrict the entry of information and adjust the unit state [18]. The loss of historical data is limited by resetting the gate *r*^*t*^. In Figures 7(b) and 7(c), the number of choreographic character series to be selected will be greatly reduced through the pruning method, so that people can select the series with the optimal conditional probability as the final transcriptome result by analyzing the optimal conditional probability of these series, denoted by *l* [19]. The application of the internal structure of GRU can be described by equations (2)–(5).

(2) $$\begin{array}{c} z^{t}=\sigma \left(W_{z}\left[h^{t-1},x^{t}\right]\right), \end{array}$$

(3) $$\begin{array}{c} r^{t}=\sigma \left(W_{r}\left[h^{t-1},x^{t}\right]\right), \end{array}$$

(4) $$\begin{array}{c} {\tilde{h}}^{t}=\tanh\left(W\left[r^{t}*h^{t-1},x^{t}\right]\right), \end{array}$$

(5) $$\begin{array}{c} h^{t}=\left(1-z^{t}\right)*h^{t-1}+z^{t}*{\tilde{h}}^{t}. \end{array}$$

${\tilde{h}}^{t}$ is the temporary hidden state at time *t*, and all *W* matrices represent the connection weights between two nodes [20]. ^*∗*^ refers to the product, that is, the elements corresponding to the matrices are multiplied, and the two multiplied matrices are required to be of the same type. *z*^*t*^ is the gating signal for the state update of the control unit, and its value range is [0, 1].

RETRACTED

For the input frame-by-frame prediction matrix *y*, CTC defines a conditional probability for any possible path *π* of length *T* on the matrix, as shown in the following equation:

(6) $$\begin{array}{c} p\left(\pi |y\right)=\prod_{t=1}^{T}y_{\pi_{t}}^{t}. \end{array}$$

*y*_*π*_*t*__^*t*^ represents the probability of predicting the action *π*_*t*_ at time *t*, counting the symbols as “aabc”. Due to individual differences of dancers, subtle differences in motion duration may lead to misalignment of consecutive movements [21]. CTC can avoid this problem. The conditional probability of *y* through the mapping function *B* and the dance notation symbol *l* is defined as the sum of the path conditional probabilities from *B* to *l*, as expressed in

(7) $$\begin{array}{c} p\left(l|y\right)=\sum_{\pi :B\left(\pi \right)=l}p\left(\pi |y\right). \end{array}$$

Σ stands for a function, and the CTC principle of path pruning using dynamic programming is shown in Figure 8 [22]. In practice, overlapping terms will increase the amount of computation exponentially, so an approximate calculation method is often used to select the most feasible motion at each time to form the optimal motion symbol sequence for the end point:

(8) $$\begin{array}{c} l^{*}\approx B\left(\underset{\pi }{\text{argmax}}p\left(\pi |y\right)\right). \end{array}$$

Therefore, by adopting the continuous motion recognition architecture of CTC, the end-to-end transition from continuous motion to continuous choreographic symbols is completed. In this step, there are no arbitrary manual alignment marks, and prior signals, such as the number of element actions [23]. Therefore, by training the model as a whole according to the loss function of CTC, the most expressive frame-by-frame fine-grained temporal characteristics can be obtained in the simulation, so that the sequence transcription of the optimal choreographic symbols is obtained for the expected CTC characteristics of the discriminative frame-by-frame dynamics in the output.

### 2.3. A Choreography Teaching Semi-supervised System Based on NNs

The motion duration labelling system supplements and improves the motion duration data under the premise of realizing the global optimization of continuous action recognition, regardless of dynamic accuracy generated by the choreography symbol sequence, so it belongs to the semi-supervised calculation [24]. The refined rendering process of continuous dance notation based on semi-supervised dynamic frame clustering is shown in Figure 8.

Figure 8 introduces the basic process of the method, in which the first half is the continuous motion recognition process, and the second half is the semi-supervised dynamic time-stamping process. First, the motion time-stamping system takes the body skeleton characteristics obtained in the identification stage as the entry, and then the k-means mobile clustering operation is used to roughly cluster the continuous motion characteristics of each frame entered. Next, smooth pooling is performed on aggregated conclusions, and the exercise capacity curve is counted. The activity markers obtained in the continuous motion judgment stage are used as the prior information of the number of clusters to accurately find the motion segmentation points, that is, the switching time points between same motions. In the end, the time of each action is obtained, and the refined production of continuous choreography is completed [25].

RETRACTED

The dynamic clustering (DC) algorithm for temporal human motion segmentation is divided into two steps, a stage of initialization and a stage of online evolution [26]. In the stage of initialization, a fixed-length window is set, and a fully connected similarity graph is constructed with the l-frame feature vectors *x*_1_,…., *x*_*t*_ in the window to roughly initialize the number of clusters. And the k-means algorithm is used to calculate the three statistical indicators of cluster center *c*_*i*_, covariance matrix Σ, and cluster radius *r*_*i*_. In the stage of online evolution, for each input frame feature vector *x*_*t*_, the algorithm calculates the minimum distance from *x*_t_ to *S*_1_, ... , *S*_k_ of the observed cluster according to (9). The equation is as follows:

(9) $$\begin{array}{c} \text{dist}\left(x_{t},C\right)=\underset{1\leq i\leq k}{\text{min}}x_{t}-c_{i}^{2}. \end{array}$$

According to the distance dist (*x*_*t*_, *C*) and the matrix Σ, the algorithm decides to assign *x*_*t*_ to its nearest cluster or to generate a new cluster. A fully connected similarity graph of *l* vertices is constructed according to l-frame feature vectors *x*_1_,…., *x*_*i*_ in the fixed-length sliding window [27]. Each vertex *v*_*i*_ corresponds to a feature vector *x*_*i*_. The connection weight *w* of the edge between two vertices *v*_*i*_ and *v*_*j*_ is defined, as exhibited in the following equation:

(10) $$\begin{array}{c} w\left(v_{i},v_{j}\right)=\text{exp}\left(-\frac{x_{i}-x_{j}^{2}}{\sigma }\right). \end{array}$$

*σ* is an adjustable parameter, and the specific normalization equation is illustrated in the following equation:

(11) $$\begin{array}{c} L=I-D^{-1/2}AD^{-1/2}. \end{array}$$

I is an identity matrix, and *D* is a diagonal matrix whose elements are defined as *D*_i,I._ A is an adjacency matrix. Then the eigenvalues of matrix *Lλ*_1_,…, *λ*_*i*_ is calculated and the number of clusters *k* is initialized, which is a commonly used method to determine the number of clusters.

RETRACTED

Although the DC algorithm can make the most fine-grained sorting for each frame, the obtained number of clusters always exceeds the expected data, and the robustness is poor. Therefore, it is necessary to pool the results of DC, to find the correct dynamic segmentation rhythm bits according to the prior information of the dynamic number obtained in the recognition framework. The process of correctly segmenting dynamic rhythm bits is shown in Figure 9.

In Figure 9, the clustering results of the previous chapter are represented as a marker sequence of length T. In a certain area (pooling window), smooth pooling is performed on the clustering results, which can not only reduce the number of clusters, but also adapt to the characteristics of continuous human motion. The time corresponding to the obtained peak is the required action split point, as shown in Figure 10.

In Figure 10(a), the peak waves are compared pair-wise, and assuming that the horizontal distance between them is greater than or equal to the minimum distance threshold, the latter is removed, so that the filtered wave peaks reach the horizontal distance exceeding the equal minimum distance threshold. In Figure 10(b), if the number of peak waves still exceeds the required number of split points at this time, the crests of the curve can be arranged from large to small according to the ability value and the degree of standing (the vertical distance between the corresponding points). Hence, the points with a relatively small capacity value and the degree of standing are removed. Here, since the minimum distance threshold is a hyperparameter, it can be tuned according to the value of the time of continuous motion and the number of element actions.

## 3. Results and Discussion

### 3.1. Results of the Ablation Experiment for Different Input Features

The results of dynamic time-stamping based on three different input features in the calculation are analyzed, as shown in Figure 11.

In Figure 11, the algorithms that use the accuracy of action time-stamping of input features to provide the 3D position characteristics of joints can achieve the maximum precision, recall rate, and the average number of repetitions, while the accuracy of dynamic time-stamping is even higher. Since the initial motion feature capture data can be used as the relative angle characteristics of joint rotation, it can accurately record the detailed signal of body motion. However, it lacks an intuitive effect, and the Euclidean distance introduced in the DC algorithm cannot measure the difference between the angle characteristic vectors very well, so the performance of dynamic time-stamping using the original data information for input is poor. Although the skeleton vector feature can represent the relative spatial position relationship between adjacent joints, compared with the absolute spatial position relationship of the joint described by the 3D position characteristics of the joint point, because the corresponding absolute spatial correlation information is lost, the distribution of the feature value is relatively uniform. That is to say, the difference in characteristics reflected by different motions is relatively small, so it will have some negative effects on the clustering process of the calculation. Therefore, the 3D position characteristics of joints are selected as the main input objects.

RETRACTED

### 3.2. Results of the Performance Test of the Action Time-Stamping Algorithm Based on Semi-Supervised Dynamic Frame Clustering

The proposed algorithm is compared with other unsupervised action segmentation algorithms used in the automatic generation architecture of traditional choreography, and the results are shown in Figure 12.

In Figure 12, mean and sacrum represent two distinct approaches to the approximate estimation of body center in the algorithm, respectively. The given action time-stamping algorithm based on semi-supervised dynamic frame clustering is described by DC. It is found that the accuracy rate of the mean algorithm is 51.26%, the recall rate is 59.41%, and the average overlap rate is 57.95%. The accuracy rate of the sacrum algorithm is 86.07%, the recall rate is 95.74%, and the average overlap rate is 80.86%. The accuracy rate of the DC algorithm is 88.77%, the recall rate is 90.23%, and the average overlap rate is 82.14%. Compared with other existing methods, the proposed algorithm achieves better action time-stamping characteristics through the action time clustering technique and semi-supervised manual segmentation of rhythm bit selection of dynamic energy curves. Optimizations are achieved in both the average accuracy of frame segmentation and the average overlap of labeled action intervals.

Based on related theories, such as deep learning (DL) and NNs, a dynamic duration time-stamping model is firstly implemented, and an automatic generation architecture for end-to-end continuous dance notation with access to temporal classifiers is provided, and the DC algorithm is introduced. Secondly, the corresponding comparison experiments are carried out on the eigenvalues selected in advance. Wang et al. proposed a DNN that is trained from scratch to generate faces directly from raw speech waveforms without any additional identity information. Their model was trained in a self-supervised manner by exploiting the naturally aligned audio and video features in the video [28]. Deissp and Liu proposed a DNN-based human pose estimation method, which outputs high-precision pose position coordinates through a cascaded DNN regressor. This method takes advantage of recent advances in DL with the advantage of being able to predict poses in a complete way [29]. Yang and Qian adopted a temporal sparse model to automatically synthesize spoken character sequences conditioned on speech signals. They proposed a system to generate a facial video using a still image of a person and an audio clip containing speech, which does not rely on any manually tuned intermediate links. This is the first method capable of generating subject-independent real-world videos directly from raw audio. Their method can generate videos with natural facial expressions such as lip movements, winks, and eyebrow movements synchronized with audio [30]. The above scholars have discussed the dance generation model from different perspectives. In the process of writing, effective theories and methods are used for reference, and the purpose is to continuously optimize and upgrade the teaching of dance choreography and promote the long-term development of dance teaching.

RETRACTED

## 4. Conclusion

To optimize the teaching of dance choreography, first, according to the framework formed by the dance notation, a dynamic duration time-stamping model is constructed. Then, based on identifying the sequence of continuous choreography symbols, the time of each main action is marked in continuous motion, and the accurate description of corresponding choreography is completed. A DC algorithm with k-means is further introduced. Next, the smooth pooling method and the specific operation process of the label sequence obtained by clustering are described. At last, the ablation test of input feature selection, and the comparison test of unsupervised automatic segmentation are carried out, and the conclusion is drawn. Comparing the proposed algorithm with other unsupervised action segmentation algorithms used in the automatic synthesis framework of traditional choreographed dance notation, it is found that the accuracy rate of the mean algorithm is 51.26%, and the recall rate is 59.41%, and the average overlap rate is 57.95%. The accuracy rate of the sacrum algorithm is 86.07%, the recall rate is 95.74%, and the average overlap rate is 80.86%. The accuracy rate of the DC algorithm is 88.77%, the recall rate is 90.23%, and the average overlap rate is 82.14%. It demonstrates that the proposed semi-supervised algorithm achieves better action time-stamping characteristics, and achieves the optimization in both the average accuracy of frame segmentation and the average overlap rate of labeled action intervals.

RETRACTED

Due to limited energy, different limbs of the body must cooperate with each other in the human movement, and focusing on only one limb is not conducive to the subsequent analysis of more complex body movement processes. In the future, the automatic formation of choreography by DL needs more in-depth research, to provide stronger technical support for the preservation and inheritance of Chinese folk dance. The semi-supervised dance teaching method is an end-to-end dance generation model, which has a certain practical value for the interaction among intelligent dance education, cross-modal dance generation and discussion, and audio-visual technology.

## Figures and Tables

**Figure 1:** Commonly used choreography. (a) Dance notation example; (b) gait; (c) leg posture; (d) arm posture.

**Figure 2:** Display of dance notation during posture conversion. (a) From the middle to the right; (b) from the middle to the bottom.

**Figure 3:** The motion capture technology in film and television products. (a) Realistic action; (b) generative action.

**Figure 4:** Skeletal node model of the human.

**Figure 5:** The framework for automatic generation of continuous dance notation by CTC.

**Figure 6:** The algorithm diagram of CNN.

**Figure 7:** Internal structure of GRU. (a) Internal structure of the unit; (b) coarse pruning; (c) fine pruning.

**Figure 8:** The refined rendering process of continuous dance notation based on semi-supervised dynamic frame clustering.

**Figure 9:** The process of correctly segmenting dynamic rhythm bits.

**Figure 10:** Search of action cut points. (a) Rough cut; (b) fine cut.

**Figure 11:** The results of the ablation experiment for different input features.

**Figure 12:** Comparison results between the action time-stamping algorithm based on semi-supervised dynamic frame clustering and other existing algorithms.

## Data Availability

The data used to support the findings of this study are available from the corresponding author upon request.
